# Expression Profile of Inflammation Response Genes and Potential Regulatory Mechanisms in Dilated Cardiomyopathy

This article has been retracted.

**DOI:** 10.1155/2022/1051652

**Published:** 2022-08-17

**Authors:** Lifeng Liang, Jiayi Sun, Tianming Teng, Lizhu Chen, Zejian Li, Zhen Zhang, Yannan Gao, Wenjuan Zhang

**Affiliations:** Department of Cardiology, Tianjin Medical University General Hospital, Tianjin, China

## Abstract

**Background:**

The inflammatory response is important in dilated cardiomyopathy (DCM). However, the expression of inflammatory response genes (IRGs) and regulatory mechanisms in DCM has not been well characterized.

**Methods:**

We analyzed 27,665 cells of single-cell RNA sequencing dataset of four DCM samples and two healthy controls (HC). IRGs among differentially expressed genes (DEGs) of active cell clusters were screened from the Molecular Signatures Database (MSigDB). The bulk sequencing dataset of 166 DCM patients and 166 HC was analyzed to explore the common IRGs. The biological functions of the IRGs were analyzed according to Gene Ontology (GO) and Kyoto Encyclopedia of Genes and Genomes (KEGG) analyses. IRG-related transcription factors (TFs) were determined using the TRRUST database. The protein–protein interaction (PPI) network was constructed using the STRING database. Then, we established the noncoding RNA (ncRNA) regulatory network based on the StarBase database. Finally, the potential drugs that target IRGs were explored using the Drug Gene Interaction Database (DGIdb).

**Results:**

The proportions of dendritic cells (DCs), B cells, NK cells, and T cells were increased in DCM patients, whereas monocytes were decreased. DCs expressed more IRGs in DCM. The GO and KEGG analyses indicated that the functional characteristics of active cells mainly focused on the immune response. Thirty-nine IRGs were commonly expressed among active cell cluster DEGs, bulk RNA DEGs, and inflammatory response-related genes. ETS1 plays an important role in regulation of IRG expression. The competing endogenous RNA regulatory network showed the relationship between ncRNA and IRGs. Sankey diagram showed that arachidonate 5-lipoxygenase (ALOX5) played a major role in regulation between TFs and potential drugs.

**Conclusion:**

DCs infiltrate into the myocardium and contribute to the immune response in DCM. The transcription factor ETS1 plays an important role in regulation of IRGs. Moreover, *ALOX5* may be a potential therapeutic target for DCM.

## 1. Introduction

Dilated cardiomyopathy (DCM) is a nonischemic heart muscle disease associated with structural and functional abnormalities. A study in Minnesota indicated that the prevalence of DCM was 36.5 per 100,000 individuals (1/2700) [1]. However, many studies have suggested that the incidence may be underestimated and may be as high as 1-in-250 to 1-in-400 based on clinical observation [2]. Cardiomyopathy was responsible for 403,000 deaths in 2010 (5.9/100,000) [3], with a 5-year mortality rate from heart failure (HF) of approximately 50% [4, 5]. A study in 1990 found that patients with HF had elevated levels of tumor necrosis factor (TNF), which was the earliest evidence of the role of inflammation in HF [6]. However, therapies that target the inflammatory response in DCM have not been well developed.

The etiology of DCM includes genetics, infections, inflammation, autoimmune disease, exposure to toxins, and endocrine or neuromuscular causes. Myocardium injury, whether from genetic or environmental sources, induces inflammation and recruitment of immune cells to the heart [7]. The innate and adaptive immune systems are activated in DCM, recruiting macrophages, mast cells, B cells, and T cells in myocardium [8], and these cells participate left ventricular remodeling and dysfunction. A subgroup analysis of the Canakinumab Anti-Inflammatory Thrombosis Outcomes Study (CANTOS) trial found that a monoclonal antibody against IL-1*β* reduced HF-related hospitalizations and mortality [9]. However, most clinical trials targeting inflammation have had unsatisfactory results. Therefore, it is important to further explore the expression of inflammatory response genes (IRGs) and possible regulatory mechanisms in DCM.

Characterization of cell-specific and regulatory mechanisms of the inflammatory response in DCM may allow for identification of novel biomarkers or therapeutic targets. We explored the expression profile of IRGs and the regulatory mechanism of DCM using bioinformatics analysis based on single-cell RNA (scRNA-seq) and bulk RNA sequencing data. Finally, we explored potential therapeutic targets and drugs for treatment of DCM.

## 2. Materials and Methods

### 2.1. Single-Cell RNA Raw Data Processing

The scRNA sequencing was performed on normal (*n* = 2) and failing (*n* = 4) human heart tissue using an Illumina NovaSeq 6000 (Table S1) [10]. The primary data of GSE145154 was obtained from the Gene Expression Omnibus (GEO) database for analysis. The information of the enrolled dataset is listed in Table 1. The R software (version 4.1.3; The R Project for Statistical Computing; http://www.r-project.org) was used for data analysis. The Seurat R package (version 3.2.1) was used to process the scRNA-seq data [11]. The MergeSeurat function was used to merge multiple datasets. The cell was filtered using the following criteria: (1) cells with <800 genes and >4000 genes, (2) cells with unique molecular identifiers (UMI) > 20000, and (3) cells with mitochondrial gene percentage > 10%. The cells were found in the same microfluidic droplet and tagged with the same barcode during single cell capture. Finally, the DoubletFinder R package was used to remove these confounders [12].

After standardized data processing, highly variable genes (HVGs) in single cells were entirely identified after adjusting for confounders using the SCTransform function [13]. Principal component analysis (PCA) was used to identify principal components (PCs) based on HVGs. The top twenty PCs were input in uniform manifold approximation and projection (UMAP) using the ElbowPlot function. Batch correction was processed based on the Harmony package (version 0.1.0) [14], and the process avoided batch effect of sample. Next, the FindNeighbors function was used to establish a shared nearest neighbor (SNN) plot based on the first twenty PCs, and the cells were clustered using the FindClusters function. The FindAllMarkers function (|logFC| > 0.25) was used to identify differentially expressed genes (DEGs) for each cluster. The single R package was used to note different cell clusters.

### 2.2. IRG Scores

Inflammatory response-related genes were obtained from the Molecular Signatures Database (MSigDB) [15], and DEGs of each cell cluster were input to identify IRGs using the MSigDB database. According to the IRG set, the AUCell package (version 1.12.0) was used for scoring each cell cluster [16]. The expression proportion of IRGs in each cell was analyzed based on the area under the curve (AUC). According to the IRG set, the threshold of active cells was analyzed using the AUCell_exploreThresholds function. We mapped the AUC score of each cell to the UMAP, and the visualization of active cell clusters was used the ggplot2 package (version 3.3.5).

### 2.3. Bulk Sequencing Data Processing

The primary data of GSE141910 was obtained from the GEO database (Table 1). DEGs were analyzed using the limma package (version 3.46.0) [17]. DEGs with |logFC| > 1 and false positive rate (FDR) < 0.05 were considered for further analysis. Finally, the ggplot2 package (version 3.3.5) was used to draw volcano and heatmap plots.

### 2.4. GO and KEGG Analyses

Gene set enrichment analysis (GSEA) was used to enrich the biological functions. It was annotated by Gene Ontology (GO) and Kyoto Encyclopedia of Genes and Genomes (KEGG) analyses [18]. GO and KEGG analyses were performed using the fgsea package. *P* value < 0.05 and normalized enrichment score (NES) > 1 were as the thresholds for significant enrichment.

### 2.5. Construction of a PPI Network

IRG-related transcription factors (TFs) were obtained from TRRUST database (https://www.grnpedia.org/trrust/). According to the STRING database (https://string-db.org/), a protein-protein interaction (PPI) network was constructed using the commonly expressed IRG-related TFs.

### 2.6. Construction of a TF Regulatory Network

Competing endogenous RNA (ceRNA) regulatory genes were downloaded from the StarBase database (https://starbase.sysu.edu.cn/). We used the igraph package to establish the noncoding RNA (ncRNA) regulatory network based on the commonly expressed IRG-related TFs.

### 2.7. Potential Drugs Targeting IRGs

The regulatory network among common IRGs, TFs, and potential drugs was established using the Drug Gene Interaction Database (DGIdb) [19], which contained interaction data for genes and drugs. A Sankey diagram was generated to show the regulatory relationships using the ggalluvial package and the ggplot2 package.

## 3. Results

### 3.1. Single Cell Transcriptomic Analysis Showed the Heterogeneity of DCM

The bioinformatics analysis was possessed using the scRNA (GSE145154) and bulk RNA sequencing data (GSE141910), and the flow chart is presented in Figure 1. After data processing and filtering of the scRNA-seq dataset, a total of 27,665 CD45+ cells were retained for further analysis. The expression profiles for each sample are shown in Figure 2(a). After normalization of gene expression and PCA, 20 PCs were imported into UMAP for visualization (Figures 2(b) and 2(c)).

We classified the cells into 23 clusters based on marker genes or the top three DEGs for known cell lineages (Figures 3(a) and 3(b)) [20]. The expression levels of marker genes and the top three DEGs are shown in the dot plot (Figure 3(c)) and the violin plot (Figure 3(d)). Then, we showed the distribution of different cell clusters in each sample (Figure 3(e)) and compared the proportion of cell clusters between DCM and healthy control (HC) samples (Figure 3(f)). The distribution of each cell cluster was different between DCM and HC groups. The proportions of dendritic cells (DCs), B cells, NK cells, and T cells were higher in the DCM group than those in the HC group, and the proportion of monocytes was lower in the DCM group than that in the HC group (*P* < 0.05).

### 3.2. IRG Scores of Cell Clusters in DCM Tissue

We obtained 4157 inflammatory response-related genes from the MSigDB database, and the common expression of cell cluster DEGs and inflammatory response-related genes was defined as IRGs (1275 genes). The expression of IRGs in different cell clusters is shown in Figure S1. To investigate the expression profile of IRGs at the single-cell level, we selected IRG sets to calculate the activity scores of each cell cluster and identified active cell populations according to the optimal threshold value (Figures 4(a) and 4(b)). Cells that expressed more IRGs had higher value of AUC than cells that expressed fewer IRGs. A total of 7176 cells had higher AUC values when the AUC value threshold was set to 0.26. These active cells were mainly DCs, colored in yellow. Finally, the analyses of GO and KEGG were applied to investigate the functional characteristics of active cell subsets. These terms of biological function were mainly associated with immune response (Figures 4(c)–4(f)).

### 3.3. Bulk RNA Analysis Showed a Characteristic Gene Profile in DCM

We obtained bulk RNA sequencing data, which included 166 patients with DCM and 166 HCs. To investigate the expression profiles, we determined DEGs between DCM and HC samples, and a total of 1049 DEGs were found, including 735 upregulated genes and 314 downregulated genes (Figures 5(a) and 5(b)). We then performed GO and KEGG enrichment analyses on the identified DEGs. Interestingly, consistent with the functional features of scRNA sequencing active cell in DCM, we found a total of 72 common pathways (Table S2), which focused on immune responses, such as immunoglobulin receptor binding (Figures 5(c)–5(f)). These data indicated that DEGs from bulk RNA sequencing shared similar pathway terms with DEGs from scRNA sequencing in DCM, which suggested a potential role for the immune response in DCM.

### 3.4. Common IRGs and Regulatory Network

We further investigated common expression of IRGs in DCM according to different datasets. The intersection among active cell cluster DEGs, bulk sequencing DEGs, and inflammatory response-related genes was defined as common IRGs (Figure 6(a)). Common expression of 39 IRGs is shown in Figure 6(b) (Table S3). To explore the transcriptionally regulated activity of common IRGs, the common IRG-related TFs were obtained from the TRRUST database. 48 TFs were identified that were associated with the common IRGs, and the intersection among the TFs, active cell cluster DEGs, and bulk RNA sequencing DEGs is shown in Figure 6(c). Nine TFs in the active cell cluster DEGs and two TFs in the bulk RNA sequencing DEGs were retained, including NFKB1, EGR1, SPI1, ETS1, HIF1A, CEBPB, ETS2, REL, JUN, STAT4, and MYB. The expression of the TFs is shown in Figure 6(d). We established a PPI network based on the common TFs using the STRING database. We found that *ETS1* probably plays an important role as a hub gene in the transcriptional regulation of IRGs (Figure 6(e)). Next, we evaluated regulation of ncRNA for common IRGs using the StarBase database. A ceRNA regulatory network of common IRGs was constructed based on the ncRNA (Figure 6(f)). The ceRNA network showed that ncRNA regulated IRGs in DCM. Common IRGs, such as *EREG*, *CREB5*, *NAMPT*, *SLC11A1*, and *THBS1*, were expressed at significantly lower levels in DCs, and this lower expression was likely facilitated by ncRNA.

### 3.5. Potential Drugs Targeted to Common IRGs

We identified candidate drugs using gene-drug interaction data from the DGIdb database based on common IRGs. A Sankey diagram was drawn to show the regulatory network among common IRGs, potential drugs, and TFs (Figure S2). *ALOX5* had the most interactions with drugs and TFs, and it was selected for additional analysis (Figure 7).

## 4. Discussion

In this study, we analyzed scRNA-seq data to characterize the distribution of immune cells and the expression profiles of IRGs in DCM. The distribution of cell clusters was significantly different between the DCM and HC groups. Twenty-three cell clusters were identified, and the proportions of DCs, B cells, NK cells, and T cells were higher in the DCM group than those in the HC group. Moreover, DCs expressed more IRGs in DCM, and active cell DEGs were primarily enriched in the immune response pathway. Our findings showed that increased active status of IRGs in DCs may play a critical role in DCM by regulating the immune response.

DCs are antigen presenting cells in adaptive and innate immunity and regulate foreign antigens and peripheral self-tolerance [21]. A study showed that the level of circulating DCs was increased in patients with DCM [22]. Accumulation of DCs was also found in the heart tissue during development of heart-specific inflammation, and MHC class II molecules were also upregulated following nonspecific inflammation [23, 24]. DCs are recruited from the circulation to myocardial tissue, which promotes inflamed injury. Heart tissue injury results in increased DC-induced recruitment of potentially autoreactive T cells that may target the heart [25]. The differentiation of naive T cell into CD4+ T cells is improved by mature DCs, resulting in an adaptive immune response [26]. According to a DC-mediated model of autoimmune myocarditis, the study found that MyD88/interleukin-1 signaling was a key factor in myocardial fibrosis [27]. In our study, we also found that the number of T cells was increased in the heart tissue of the DCM group. In contrast, a study showed that the number of DCs was reduced in heart biopsies of symptomatic patients with DCM patients, which was associated with poor short-term outcomes [28]. The role of DCs in the pathophysiology of DCM is controversial, and the potential mechanisms require further study.

We further analyzed bulk RNA sequencing data from DCM human heart tissue. The results showed that DEGs from bulk RNA sequencing shared similar functional characteristics with the DEGs in the scRNA sequencing data analysis and were mainly associated with the pathway of immune response. These results suggested that the identified IRGs were important signatures of DCM. Inflammation-related genes are critical to immune stimulation and infiltration of immune cells [29]. Previous study found that expression profiles of heart tissue showed that failing and nonfailing heart expressed different genes related to immune responses, and the difference was also found between ischemic HF and nonischemic HF [30]. PPI network revealed a cluster of significant differently expressed proteins related to the immune response in the pathogenesis of disease progression in DCM. Furthermore, *ETS1* may be a hub gene involved in regulation of IRGs. The regulation of ncRNA in common IRGs further demonstrated that the immune response may be a key factor in DCM. Functional ncRNA plays a role in regulatory mechanisms of HF, leading to ventricular remodeling, hypertrophy, and myocardial apoptosis. A recent study indicated that the suppression of miRNA-152-3p improved the expression of *ETS1*, promoting the development of HF [31].

Finally, we found that *ALOX5* participated the regulation of IRG-related TFs and the actions of potential drugs. Common IRG-related TFs such as EGR1 and NKKB1 have been shown to regulate the expression of *ALOX5* [32]. 5-Lipoxygenase is a subtype of human *ALOX* family, which promotes generation of lipid peroxides, resulting in excessive lipid peroxidation of phospholipids [33]. Excessive lipid peroxidation of the plasma membrane can result in membrane rupture and cell death, which leads to increased inflammation through release of damage-associated molecular patterns [34]. 5-Lipoxygenase also participates in the biosynthesis of leukotrienes (LTs), which are major mediators of inflammation in human diseases, such as asthma, atherosclerosis, Alzheimer's disease, and diabetes [35]. Upregulation of *ALOX5* has been shown to induce LT production in human DCs treated with lipopolysaccharide [36]. Moreover, overexpression of *ALOX5* accelerated myocardial injury and cardiac dysfunction in a sepsis mouse model [37]. A study showed that inhibition of *ALOX5* improved functional recovery in a rat model of cerebral ischemia [38]. Furthermore, atorvastatin, a commonly used drug, induced 5-lipoxygenase phosphorylation, which increased production of anti-inflammatory mediators in atherosclerosis [39]. Therefore, *ALOX5* may be a therapeutic target for treatment of DCM.

In summary, our study indicated that DCs may infiltrate heart tissue, and IRGs of DCs may contribute to regulation of the pathway of immune response in DCM. Furthermore, we identified potential regulatory mechanisms of IRGs in DCM. Moreover, *ALOX5* may be a therapeutic target for DCM. The scRNA-seq methods provided an additional dimension of transcriptional information of individual cells relative to bulk population of cells. Our analysis associated with scRNA and bulk RNA sequencing data to explore the heterogeneity in different cell cluster of DCM. However, our study suffered from the following limitations. First of the sample size for patients with DCM was small. The limited sample size may have prevented the capture of the characteristics of DCM, as DCM is a heterogeneous disease. In addition, immune cell infiltration, IRGs expression, and the regulatory mechanisms of DCM require further validation *in vivo*.

## 5. Conclusion

We evaluated the IRG expression profile of DCs and identified possible IRG-related regulatory pathways in DCM. DCs are recruited into the heart tissue and contribute to the regulation of immune response in DCM, as evidenced by bioinformatic analysis using scRNA and bulk RNA sequencing data. The transcription factor ETS1 may play an important role in regulation of IRG expression. Moreover, *ALOX5* may be a potential therapeutic target for DCM.

## Figures and Tables

**Figure 1:** Flow chart of bioinformatics analysis. Abbreviation: scRNA-seq: single cell RNA sequencing; MSigDB: Molecular Signatures Database; DEGs: differentially expressed genes; IRGs: inflammatory regulatory genes; GO and KEGG Gene Ontology and Kyoto Encyclopedia of Genes and Genomes; PPI: protein–protein interaction network; ceRNA: competing endogenous RNA.

**Figure 2:** Single-cell raw data quality control. (a) The gene number, molecular number, and the proportion of mitochondrial genes in each sample. n_Feature represents the number of genes in each cell. n_Count represents the number of molecules in each cell. (b) Elbow graph of PCA. (c) UMAP dimensional plot after adjusting for batch effects.

**Figure 3:** scRNA analysis reveals the heterogeneity of immune cells in DCM. (a, b) The UMAP plots represent 23 cell clusters from six samples (four DCM and two HC). (c) Violin graphs show the marker genes in 23 distinct cell types. The width of violin plot is related to the frequency of cells with relevant gene expression level. (d) Dot graphs show the expression of the top three DEGs for each cell type. The colors of dots represent average expression, and the sizes of dots represent the average percent of cells that expressed the DEGs. (e) Bar graphs show the proportion of cell clusters in different samples. (f) The comparison of each cell type between DCM and HC. Data were analyzed according to chi-square test. ^∗∗∗∗^*P* < 0.0001, ^∗∗∗^*P* < 0.001, ^∗∗^*P* < 0.01, and ^∗^*P* < 0.05. ns: not significant.

**Figure 4:** The cell activity scores of cell clusters. (a) The score of the IRG set. The threshold was 0.26, and the active scores of 7176 cells exceeded the threshold. (b) The UMAP dimensional plot according to the active score of each cell cluster. (c–f) GO and KEGG pathway enrichment analyses of DEGs in high and low active cell clusters. GSEA for pathways in KEGG includes systemic lupus erythematosus, cytokine–cytokine receptor interaction, primary immunodeficiency, and ribosome. GSEA for molecular function in GO includes MHC class II receptor activity, immunoglobulin binding, IGG binding, immunoglobulin receptor binding, and signaling adaptor activity. GSEA for biological process in GO includes T cell activation via T cell receptor contact with antigen bound to MHC molecule on antigen presenting, B cell homeostasis, and endogenous peptide antigen via MHC class I tap independent. GSEA for cellular component in GO includes MHC class II protein complex, large ribosomal subunit, MHC class I protein complex, immunoglobulin complex, and immunoglobulin complex circulating.

**Figure 5:** DEGs between DCM and HC from bulk sequencing data. (a) Volcano plot shows DEGs between DCM and HC groups. (b) Heatmap shows the expression of DEGs between DCM and HC groups. (c–f) GO and KEGG pathway enrichment analyses of DEGs from bulk sequencing data. GSEA for pathways in KEGG includes renin angiotensin system, gap junction, pathogenic Escherichia coli infection, and complement and coagulation cascades. GSEA for molecular function in GO includes immunoglobulin receptor binding, antigen binding, organic acid binding, extracellular matrix structural constituent, and flavin adenine dinucleotide binding. GSEA for biological process in GO includes acute phase response. GSEA for cellular component in GO includes T cell receptor complex, collagen trimer, immunological synapse, immunoglobulin complex circulating, secretory cranule membrane, polymeric cytoskeletal fiber, and tertiary granule membrane.

**Figure 6:** The characteristics of common IRGs and regulatory network. (a) The intersection among bulk RNA sequencing DEGs, active cell cluster DEGs, and inflammatory-related gene set. (b) The expression of the common IRGs. (c) The intersection among common IRG-related TFs, active cell cluster DEGs, and bulk RNA sequencing DEGs. (d) The expression of common TFs. (e) The PPI network of common IRG-related TFs. (f) The regulatory network of noncoding RNA in common IRGs.

**Figure 7:** Regulation of TFs and potential drugs by common IRGs. ALOX5 had the most interactions with drugs and TFs.

**Table 1:** The datasets of the study.

Dataset	Type	Platform	Sample size (HC/DCM)
GSE145154	scRNA	GPL24676 Illumina NovaSeq 6000 (Homo sapiens)	2/4
GSE141910	Bulk RNA	GPL16791 Illumina HiSeq 2500 (Homo sapiens)	166/166

scRNA: single-cell RNA; DCM: dilated cardiomyopathy; HC: healthy control.

## Data Availability

Data are available in a public, open access repository.

## Supplementary Materials

Supplementary Materials Figure S1: the expression of IRGs in different cell clusters. Figure S2: the regulation network of common IRGs to TF and potential drugs. The Sankey diagram was drawn to demonstrate the regulatory network among common IRGs, potential drugs, and TF. *ALOX5* had the most interactions with drugs and TF. Table S1: the information of samples. Table S2: common pathways in scRNA and bulk RNA data. Table S3: common IRG list.
